RETRACTED

# Public Art and Space Environment Design Using Genetic Algorithm-Guided 3D Virtual Reconstruction

**DOI:** 10.1155/2022/2193950

**Published:** 2022-09-09

**Authors:** Man Luo

**Affiliations:** School of Art and Design, Shanghai University of Engineering Science, Shanghai 201620, China

## Abstract

Public art plays a crucial role in influencing the development of the urban space environment by embodying the spiritual outlook and cultural heritage of a city. The research status and development trend of contemporary public art and space environment design are introduced in this article. In this essay, the relationship between public art and the environment of public spaces is examined in terms of type, status quo, and impact. The requirements of the virtual process are then thoroughly examined through the practical application of various collaborative software based on the actual needs of 3D virtual reconstruction. In parallel, a genetic algorithm-based optimization design scheme for the space environment is proposed. Numerous experiments are conducted to confirm the viability of this method. The efficiency of this algorithm, according to experiments, is very high, reaching 94.87 percent. The scores of the residents are also good as a result of this article's design. This demonstrates the validity of this approach. The study of public art and urban space environment design is expected to contribute positively to the growth of the city.

## 1. Introduction

Public art plays a significant role in urban planning. Public art is a city's calling card for growth, representing its cultural heritage and spiritual outlook, and it is essential to determining the character of the urban environment [1]. Public art has an unavoidable social and cultural history if we are to judge by its emergence. People's material and cultural lives have never been richer thanks to the global economy's quick development. People are more aware of their local city as well as the interactions and coordination between locals and their surroundings. Additionally, public art acts as a medium for dialogue between individuals, groups of individuals, and the broader community [2]. Being a public, democratic, and open art, it can reflect the needs of the entire society as well as social issues and public sentiment. In the modern era, urban public art has reached a stage of full development. However, the globalization of economy and culture has also brought many problems to public art design: urban public art tends to be one side of thousands of cities; there are only a few people who plan and decide on public art, which lacks publicity; and designers lack understanding of artistic language and publicity. From the perspective of environmental development, the demand for resources today is unprecedented [3]. The excessive demand for resources intensifies the contradiction between man and the environment. The existence of public art can just be used to alleviate this contradiction. How to meet the living relationship and demand between nature and people, let public art take social responsibility, and introduce public art's humanistic concern for space environment into environmental space is the most urgent task we are facing [4]. The economic level is only one factor in the success of a city's development, but it cannot cover all of them. The cultural heritage of a city is a powerful driving force for the city's long-term survival and development. Therefore, the design of public art and space environment is particularly important [5]. The research of public art and urban space environment design is of positive significance to promote the development of the city. Many charming cities are not only because they have a long history and profound cultural heritage, but also because they have many attractive external spaces.

RETRACTED

Public participation is the cornerstone of public art life, and public art serves the public. Designers can only comprehend the current situation and issues pertaining to the development of Chinese contemporary public art by furthering their analysis and understanding of the issues [6]. This will also allow them to have a deeper understanding of many factors that affect the public space and the public. Making public art more pervasive in people's daily lives can increase public understanding of it, improve the precision with which it expresses space environment culture, pique public interest in participating in it, and lay a solid foundation for its future development. At the same time, it can encourage the peaceful coexistence and shared development of the human environment in both the social and natural spheres [7]. The appearance of virtual reality is the result of in-depth research on “human factors” in network, multimedia, and other technologies. It provides a new direction and space to study virtual reality effects from the perspective of users' psychology and sensory feelings. 3D reconstruction is a very important research topic in computer vision, computer graphics, virtual reality, and other fields [8]. Using 3D reconstruction technology, computer graphics system can not only realize design and drawing but also directly process the drawing results. Based on the basic characteristics of virtual reality and its application in the field of design art, this article discusses public art and space environment design based on 3D virtual reconstruction technology. Its innovations are as follows:

1. In this article, the related research and technical methods of 3D virtual reconstruction, target recognition, and parametric modeling are discussed, and the existing problems are pointed out and improved. The information extraction and integration method of engineering drawings adopted in this article overcomes the difficulties of 3D reconstruction of architectural drawings and completes the overall 3D reconstruction. In addition, the step-by-step and hierarchical automatic recognition method in this article can not only make full use of the convenience and efficiency of computer automatic image reading but also insert manual interaction after each step to correct errors and omissions in automatic recognition in time and prevent errors from spreading to subsequent processing results.
2. This article proposes a space environment optimization design scheme based on a genetic algorithm in response to the current situation where the general recognition rate and recognition accuracy of conventional methods are not optimal. Numerous experiments are conducted to confirm the viability of this method. The algorithm presented in this article is effective and trustworthy, according to experiments.

RETRACTED

## 2. Related Works

Scognamiglio and Garde proposed an automatic reconstruction system based on a knowledge system from aerial image sequences, which needs to provide a two-dimensional GIS map and an image sequence of the reconstructed area [9]. Wang et al. summed up four principles that public art should follow in the process of design and creation: ① the principle of necessity for public art to exist in urban public space, ② the principle of common development of various types of public art, ③ the principle of humanistic concern for public art, and ④ the principle of uniqueness of public art [10]. Zhou's 3D display and roaming of building structures based on OpenGL discussed the method of realizing 3D display and roaming of building structures with OpenGL [11]. Jaganmohan et al. first extracted approximate building outlines from the data, which were fitted by splicing multiple rectangles, then connected and optimized adjacent rectangles to obtain complete and complex building outlines, and finally extracted elevation information to complete 3D city modeling. This method has achieved good results in the reconstruction of complex buildings [12]. Sha et al. need to do a more in-depth and comprehensive research on the current status of the public art design. Establishing a theoretical system of public art, cultivating public art design talents, and strengthening the research on the humanities and natural environment of public spaces are important tasks of current public art [14]. Li and Hou proposed a method for building extraction and 3D reconstruction based on the LiDAR point cloud. This method can not only reconstruct simple and regular buildings but also reconstruct buildings with complex roof planes and irregular structures [15]. Allahyar and Kazemi had made in-depth research on application system design and implementation, overall identification method, coordinate system identification and global integration, table identification and parameterization method, and engineering drawing object identification method [16]. Sun et al. collected and sorted out some materials on public art and its related concepts “public” and “public space,” as well as the origin and history of public art, focusing on the inseparable relationship between them. [17]. Wang proposed a 3D reconstruction technique of regional buildings based on radar data and aerial images [18]. The method firstly creates a grayscale elevation map based on radar data, then extracts building edges from it, extracts building height data from radar data, extracts texture from aerial photo images, and finally generates a 3D model.

RETRACTED

The accuracy and recognition rate of traditional methods are generally not the best. The relationship between public art and the environment of public spaces is examined in this article through an examination of the different types, the current state, and its impact on the environment. The requirements of the virtual process are then thoroughly examined through the practical application of various collaborative software, based on the actual needs of 3D virtual reconstruction. Additionally, the information extraction and integration method of engineering drawings used in this article solves the problems associated with the 3D reconstruction of architectural drawings. Experiments demonstrate some reliability for this method.

## 3. Methodology

### 3.1. Application of 3D Virtual Reconstruction in Public Art and Space Environment Design

Public art has recently grown in importance as a component of urban environmental design. Being a public, democratic, and open art, it can reflect the needs of the entire society as well as social issues and public sentiment. Urban public art is essential to the development of cities. Public art is evolving at an increasingly rapid rate due to the ongoing growth of economic and spiritual civilization. Public art's central theme is public sex. Due to differences in cultural background, social class, occupation, gender, age, and a variety of other factors, people's understanding and cognition of the concept of public art vary greatly precisely because of its publicity. The vitality of public art itself, however, may lie in the existence of such diverse opinions and debates regarding it. Public art can be thought of as the artistic welfare of the people, and equal sharing of rights is determined by publicity. The public can share, express themselves artistically, congregate and unwind, and interact with one another in this space because it was created based on the wishes of the majority of people and because of its spatial characteristics. Public art is a significant way to increase the diversity of urban culture and disseminate cultural knowledge to the general public, and it can help shape a city's distinctive cultural traits and spiritual outlook. However, modern public art should not only satisfy the urban image construction or simply beautify the urban public space but also try to create a higher quality and sustainable urban living environment while satisfying them. At present, the main problem that affects the development of public art is that the public's understanding and cognition of public art is insufficient, and people have not formed their awareness of the public art system at the level of consciousness. This directly leads to the lack of public attention and participation in public art, thus restricting the healthy and all-around development of public art. Any design is inseparable from the two themes of aesthetic function and practical function. As the functional attribute of public art must consider the aesthetic function of the public, it is inseparable from the public. If artists do not consider their works from the perspective of the public, works created by self-entertainment and narcissism cannot be regarded as public art.

RETRACTED

The design of public art and space environment is more widely combined with modern digital media technologies such as advertising, animation, games, and music and has achieved good performance results. Urban public space is the exhibition stage of public art, and the establishment and completion of public art must be carried out in this space. The necessary condition of public participation is to define and clarify the service object and existence value of public art, and it is the foundation that distinguishes public art from other forms of art. The change in the nature and function of urban public space will inevitably lead to a change in public art style, and the form of public art is constantly changing and accumulating with the historical connotation of urban social form and public space. The development of a large number of advanced technologies such as human-computer interaction technology and artificial intelligence (AI) technology [19, 20] of digital media technology has expanded the functional range of digital media technology, and at the same time, people can use digital media technology to make ideas possible and realize the leap from ideal to reality [21]. Among them, virtual reality technology breaks people's inherent thinking concept, realizes landscape space in a virtual world, and brings users into an immersive landscape design experience space through high simulation, user participation, scene simulation, and real-time calculation. This space expands the designer's thinking, creates rich and novel design methods, and exerts the imagination of traditional landscape planning and design to the extreme. 3D reconstruction is a very important research topic in computer vision, computer graphics, virtual reality, and other fields. Modeling is the model of a scene component, which is the basis of rendering, and the subsequent operations are recreated based on the model. In practical work, there are two commonly used modeling bases, namely modeling based on CAD drawings and modeling based on pictures. With the rapid development of the digital city and the continuous expansion of the application field of urban 3D space model, the demand for 3D models of public art and space environment design is increasing. Virtual landscape is the differentiation and integration of human thoughts and dreams and the description and portrait of human thoughts and ideas. The powerful advantages and unlimited development prospects of the virtual landscape can only be reflected through its extensive and in-depth application.

3D reconstruction refers to the establishment of 3D models corresponding to real objects with a certain level of detail in the digital virtual environment. The 3D reconstruction process includes two stages: ① the acquisition of building basic data and ② 3D model construction. Public art serves the public, and public participation is the foundation of public art life. In the process of design and implementation, first, we should encourage the public to actively participate and improve the owner's consciousness. Second, we can popularize the public's awareness through newspapers, Internet, television, libraries, art galleries, and other channels to improve the public's aesthetic quality. The design of public art and space environment refers to the overall consideration, design, and treatment of surrounding environmental elements through the virtual simulation and real-time interaction of 3D virtual reconstruction technology in the whole system design process so that the landscape, natural environment, and people's living environment are in harmony and mutual echo, and the landscape subject is more scientific and beautiful, and improve its overall artistic value and cultural value and meet people's emotional needs to the greatest extent. In many cases, we may have obtained data such as contour and height before 3D reconstruction, so it is easy to exclude the acquisition of basic data from the 3D reconstruction system. However, in fact, the acquisition of basic data often costs a lot of manpower, financial resources, and time. The 3D modeling method mainly consists of two steps: one is the generation of global contour lines, and the other is the generation of the 3D plane. AutoCAD is favored by users because of its powerful function and easy operation. It is widely used in mechanical design, architectural design, urban planning, and other fields. In the production of public art and space environment design renderings, you can use this software to draw the plan and elevation of garden design. Parametric technology refers to a kind of computer-aided design technology, in which parameters are related to geometric shapes, and the characteristics of geometric shapes can be controlled by adjusting parameter values. Parameterization technology includes three types, namely method based on grammar rules, method using mathematical model, and method combining artificial intelligence.

RETRACTED

### 3.2. Public Art and Space Environment Design

Judging from aesthetics, the first goal of public art and space environment design is to improve the aesthetic feeling of living environment. From the perspective of life experience, it is to improve the living environment, delight the body and mind, and improve the quality of life. From the design point of view, public art and space environment design is a process of seeking a variety of landscape composition and collocation forms, finding new combination ways, changing the existing life pattern, optimizing life, and putting forward a new way of life. Public art and the surrounding environment are not only exhibited from one perspective but also work in harmony with other structures to create a larger spatial setting. This includes both man-made and natural landscapes. In order to develop harmony between environmental protection and buildings, three-dimensional greening technology can be applied in a variety of buildings. In addition, if the public art and space environment design does not highlight the characteristics of the city, then the significance of public art and space environment design will be lost. When developing public art and space environment design, we should make good use of the excellent cultural resources of the city. In the process of making virtual renderings of public art and space environment design, computer software only plays the role of a tool. How to use this tool to create and express one's artistic concepts depends entirely on the creator himself. Therefore, there is no fixed and necessary sequence for making renderings, but there is a relatively scientific process when using computer software to make renderings. 3D modeling is a common modeling method in rendering. Based on 3D virtual reconstruction technology, this article introduces target recognition technology and parametric modeling technology, and through the reconstruction and integration of the top-level framework and the improvement and innovation of the bottom-level technology and methods, a set of low-cost and high-efficiency popular solutions for designing the 3D virtual reconstruction of public art and space environment are formed.  Figure 1 is the modeling flow chart.

RETRACTED

In 3DS MAX software, each modeling method corresponds to several series of specific tools. For example, the tools in the Geometry Creation Panel can create simple geometry commonly used in rendering, while the 2D linear creation tools can create the cross section of complex objects in a 2D linear way and then transform them into more complex 3D models by modifying commands. Public space is a place to provide recreational activities for residents. As a result, during the design phase, it is important to consider the range of residents' activities and the nature of their entertainment. Integrating public art practice into the design process will maximize the value of public art spaces and draw attention to the allure of art in design. The fuzzy evaluation method is employed in this study to gauge how satisfied locals are with the pedestrian street and square. The evaluation factor set in this article consists of 12 elements, including the variety and accessibility of the activities. Based on the evaluation elements, the ratings are classified into five groups, ranging from very satisfied to very unhappy. The weight value is utilized to compute the final evaluation result in addition to determining the degree of membership of the evaluation factors and the membership link between the evaluation factor set and the grade.

According to the relevant algorithm rules, feature calculation refers to the calculation of each primitive's spectrum, texture, shape, geometric relationship, spatial topological relationship, hierarchy, and other features one at a time. The results are saved in the data structure contained within the primitive. The comparative sorting method is used in this article to choose the ten evaluation factor set components that are most crucial, after which they are sorted and scored. Each factor's weight is calculated by dividing its percentage by the sum of all factor scores:

(1) $$\begin{array}{c} w_{j}=\frac{\sum_{i=1}^{n}k_{ij}}{\sum_{j=1}^{m}k_{ij}}, \end{array}$$

where *n* represents the number of evaluations, *m* represents the number of evaluation factors, and *w*_*j*_ represents the weight of the *j*th evaluation factor.

RETRACTED

The architecture of public art spaces should conserve biological diversity in order to accurately depict the natural and ecological characteristics of urban public art spaces. As a result, the actual urban ecological situation should be considered while designing public art places. Based on residents' satisfaction with the landscape space at the entry and departure of architectural landscape, parking lots, and other public facilities, the size and space of architectural landscape are optimized in this study. The analytical hierarchy process (AHP) is used to determine the different architectural landscape kinds, and the judgement matrix for the index layer is constructed along with its weight value. The weight judgement matrix of the index layer can be expressed as follows:

(2) $$\begin{array}{c} W=\left(0.382,0.016,0.036,0.018,0.206,0.121,0.169,0.037,0.045\right). \end{array}$$

A comprehensive analysis of the weights of public facilities in landscape space such as green belts, seats, and parking spaces shows that the final weights are 0.418, 0.121, and 0.236 respectively.

The initial component contour coordinates are based on the local coordinate system of the drawing, which may have different starting points and rotation angles, and these local coordinate system contours must be transformed into global coordinate system contours. Two different grid points (*P*_0_, *Q*_0_) and (*P*_0_, *Q*_*n*_) are taken in the local coordinate system, where (*P*_0_, *Q*_0_) is the origin of the local coordinate system. The corresponding local coordinates are divided into

(3) $$\begin{array}{c} \left(u_{0},v_{0}\right),\left(u_{1},v_{1}\right). \end{array}$$

**Assumption 1 .**

(4) $$\begin{array}{c} \text{len}=\sqrt{{\left(u_{1}-u_{0}\right)}^{2}+{\left(v_{1},v_{0}\right)}^{2}}. \end{array}$$

Then,

(5) $$\begin{array}{c} \text{Sin}\theta =\frac{\left(v_{1}-v_{0}\right)}{\text{len}}\text{ Cos}\theta =\frac{\left(u_{1}-u_{0}\right)}{\text{len}}. \end{array}$$

If the global coordinate of (*P*_0_, *Q*_0_) is (*x*_0_, *y*_0_), the transformation matrix is

(6) $$\begin{array}{c} M=\left[\begin{array}{c} \text{Cos}\theta -\text{Sin}\theta -x_{0}\text{Cos}\theta +y_{0}\text{Sin}\theta \\ \text{Sin}\theta -\text{Cos}\theta -x_{0}\text{Sin}\theta +y_{0}\text{Cos}\theta \\ 0\;01 \end{array}\right]. \end{array}$$

Each contour vertex's global coordinates are determined using the matrix. When raster data are vectorized, vector arcs are created along the borders of adjacent areas, and by connecting the connected arcs, closed vector polygons are created to enclose raster areas. Although the final vector polygon has only basic features, since pixels are used throughout the entire vectorization process, this process falls under the category of pixel-level processing. The system's foundational step, vectorization, will lay the groundwork for analysis and processing based on primitives. The prices of different construction facilities are included in the objective function of construction cost and can be expressed as follows:

(7) $$\begin{array}{c} \text{Min}\cos\;t=\sum_{1\leq j\leq n}a_{j}\times \Delta X_{j}, \end{array}$$

where cos  *t* represents the input cost of architectural and landscape facilities, *a*_*j*_ represents the price of architectural and landscape facilities, and Δ*X*_*j*_ represents the number of architectural and landscape facilities. In a comprehensive consideration, the resident satisfaction function can be expressed as

(8) $$\begin{array}{c} \text{Max}S=\sum_{1\leq j\leq n}W_{j}\times \left(X_{j}+\Delta X_{j}\right)\Delta X_{j}\in E, \end{array}$$

where *S* represents satisfaction, *W*_*j*_ represents the weight value of facilities, *X*_*j*_ represents the number of landscape facilities installed in the building, and Δ*X*_*j*_ represents the number of added landscape facilities. The genetic algorithm process is shown in Figure 2.

RETRACTED

The values of the crossover probability *P*_*c*_ and the mutation probability *P*_*m*_ will rise in the adaptive genetic algorithm if the population's fitness is in a substantially concentrated state. The levels of *P*_*c*_ and *P*_*m*_ will fall, however, if the population's fitness is in a more dispersed state. The following two equations determine how the two parameter probabilities automatically modify their values:

(9) $$\begin{array}{c} P_{c}=\left\{\begin{array}{cc} \frac{k_{1}\left(f_{\max}-f^{\prime }\right)}{\left(f_{\max}-f_{\text{ave}}\right)}, & f^{\prime }\geq f_{\text{ave}},\\ k_{2}, & f^{\prime }<f_{\text{ave}}, \end{array}\right.\\ P_{m}=\left\{\begin{array}{cc} \frac{k_{3}\left(f_{\max}-f\right)}{\left(f_{\max}-f_{\text{ave}}\right)}, & f\geq f_{\text{ave}},\\ k_{4}, & f<f_{\text{ave}}, \end{array}\right. \end{array}$$

where *f*_max_ represents the highest fitness, *f*_ave_ represents the average fitness, *f*′ represents the fitness of the individual with relatively high fitness among multiple crossover individuals, and *f* represents the individual fitness that produces variation, and

(10) $$\begin{array}{c} 0<k_{1},k_{2},k_{3},k_{4}\leq 1. \end{array}$$

It is important to emphasize the landscape experience, improve the appreciation of the public art space environment, and incorporate the “humanistic spirit” into it. Public art space designers should consider all aspects according to residents' physical and psychological conditions and design personalized places that meet people's needs. Generally speaking, the materials required for the production plan should be produced and adjusted in accordance with the external effects depicted in the designed drawings, and the renderers and designers should keep in regular and timely contact throughout the production process. Data preprocessing techniques include cloud removal, spectral normalization, image fusion, mosaicing, geometric correction, registration, and image cropping. Its goal is to ensure that the remote sensing image data being processed satisfy the criteria for postprocessing and analysis, as well as the efficacy and accuracy of the results. This article combines different framing transformation techniques so that the viewer can easily move forward, backward, left, right, up, down, and rotate in order to view the space environment design that is depicted in the scene from all angles and directions. The images produced by 3DS have a lot of flaws for a variety of reasons. Postprocessing is required to address these deficiencies. However, in order to increase productivity, we typically choose to create them later because many effects are challenging to create in 3DS MAX but simple to create in Photoshop.

RETRACTED

## 4. Result Analysis and Discussion

Urban public spaces are improved by public art, but while improving and beautifying public spaces, improper planning, unfounded design, and inappropriate planning can also ruin a formerly wonderful public space. Public space in a city can be impacted positively or negatively by the planning and design of public art. The model offers the system's design blueprint by condensing and simplifying reality. The model can incorporate not only specific plans but also high-level ideas and big-picture plans from the design world. A good model includes the important components that have a widespread impact while ignoring the minor components that have no bearing on the stated abstract requirements. Various models based on various aspects can be used to describe each system. VH-RecQS, as a new generation of map reading and calculation software, overcomes the shortcomings of traditional calculation software. It can automatically identify the building drawings to calculate the engineering quantity, which is fast and efficient, accurate and reliable, easy to operate and easy to learn, and the system has excellent stability. This chapter makes an experimental analysis of the design method of public art and space environment based on 3D virtual reconstruction. In the experiment of this chapter, we selected a high-resolution remote sensing image of QuickBird in a certain area with a spatial resolution of 0.8 meters, including blue, green, and red bands, as the experimental object. First, due to the limitation of spatial resolution, the interference of noise, and the error caused by the discretization of raster data, the boundary of vector space data generally presents irregular silver teeth. In order to weaken the data and improve the compression accuracy, this article recommends the method of iterative Gaussian filtering to smooth the vector graphics. The convergence of the algorithm is shown in Figure 3.

RETRACTED

Public art cannot let people directly participate, which has dampened the enthusiasm of public participation. The public cannot find or realize the intersection of public art and itself and can only ignore or even ignore public art, and the distance between public art and the public is getting farther. For a good design, the simulation of the interior landscape of the building needs to highlight the sense of light, the beauty of curves, and the sense of volume of space, and the form is enclosed with each other. The foundation is located on a connected foundation slab, and the roof steel structure is covered with a double-layer membrane structure, which is light, meticulous, and varied. Greening should also follow the design idea of being separated from the steel structure but matching each other into a landscape. After reading the information in the drawings, we should first analyze the underlying objects; merge overlapping lines, connected arcs, and connected solid bodies; analyze the relationship between lines; and preliminarily identify the steel bar labeling strings represented by various forms of character sets. In order to verify the advantages of this method in efficiency and accuracy, we made further comparative experiments.  Figure 4 shows the efficiency comparison results of different methods, and Figure 5 shows the relationship between cost spacing and relative segmentation accuracy.

Through the interactive function provided by the recognition and system, the basic component information such as coordinate system, column, wall, beam, and plate can be extracted from the diagram, and then the components can be analyzed and the relationship between them can be established. The facade of the main body of the model shall be sealed by walls to avoid light scattering or light leakage of glass materials; avoid double surfaces between walls to prevent rendering from breaking surfaces; collapse a series of model elements into an object and delete the unseen to simplify the model—the same material object collapses into an object so that there is no two-dimensional line; and map before collapsing and confirm the modification before collapsing. The optimization in this article refers to the processing of the boundary of vector graphics according to certain rules so as to make it within a certain precision range. On the one hand, it can make its shape closer to the real contour or meet specific application requirements; on the other hand, it can effectively reduce the amount of node data.  Figure 6 shows the comparison of compression time consumption of equal processing rate under different threshold conditions, and Figure 7 shows the comparison of treatment rates under different threshold conditions.

RETRACTED

Public art and urban public space have been developed, revised, and improved constantly as the general public has grown to be the dominant segment in society. An investigation found that openness, diversity, and convenience can all be utilized as evaluation markers. Openness is the idea of open architectural space, diversity is the idea of a variety of activities, and convenience is the idea of public utilities being easily accessible.  Table 1 displays the various evaluation variables for squares and pedestrian streets together with their attention levels, and Table 2 displays the satisfaction of the landscape area that was optimized.

It can be seen that after the design of this article, the rating data of residents are at a high level. The 3D display function of VH-RecQS software can not only preview the structure of the whole building but also reflect the recognition efficiency instantly and intuitively. It provides a good check method for the recognition function of software and improves the efficiency of software recognition.

## 5. Conclusions

Public art is an essential visual art image in a city because it can record, contain, and inherit the history and culture of the place. Urban public art and space environments should be designed so that they fully reflect a city's style, historical context, and cultural connotations in addition to meeting the basic requirements of providing urban public cultural services. The research status and development trend of contemporary public art and space environment design are introduced in this article. In this essay, the relationship between public art and the environment of public spaces is examined in terms of type, status quo, and impact. The related research and technical methods of target recognition, parametric modeling, and 3D virtual reconstruction are also discussed at the same time, and the problems that currently exist are identified and corrected. The requirements of the virtual process are then thoroughly examined through the practical application of various collaborative software, based on the actual needs of 3D virtual reconstruction. The challenges of 3D reconstruction of architectural drawings are overcome by the information extraction and integration method of engineering drawings used in this article, which also completes the overall 3D reconstruction. The step-by-step and hierarchical automatic recognition method in this article can also incorporate manual interaction after each step to correct errors and omissions in automatic recognition in real time and prevent errors from spreading to the results of further processing. This way, it is possible to fully utilize the efficiency and convenience of computer automatic image reading. The efficiency of this algorithm, according to experiments, is very high, reaching 94.87 percent. The scores of the residents are also good as a result of this article's design. This demonstrates the validity of this approach. This article still has some flaws, though, and they require further study. The introduction of the parallel cluster method is another highly effective way to increase the effectiveness of target recognition, in addition to optimizing the recognition method itself. It offers countless options for the effective identification of enormous amounts of remote sensing data and is an extremely important research area.

RETRACTED

## Figures and Tables

**Figure 1:** Modeling flow chart.

**Figure 2:** Flow chart of genetic algorithm.

**Figure 3:** Convergence of algorithm.

**Figure 4:** Efficiency comparison results of different methods.

**Figure 5:** Relationship between cost spacing and relative segmentation accuracy.

**Figure 6:** Comparison of equal processing rate compression time consumption under different threshold conditions.

**Figure 7:** Comparison of treatment rates under different threshold conditions.

**Table 1:** Different degrees of attention of evaluation factors of squares and pedestrian streets.

Serial number	Evaluation factor	Square	Pedestrian street
1	Space security	0.066	0.069
2	Space privacy	0.072	0.074
3	Greening rate	0.179	0.161
4	Color diversity	0.085	0.079
5	Convenience of public facilities	0.257	0.245
6	A broad sense of vision	0.078	0.080
7	Leisure atmosphere	0.171	0.192
8	Individualization degree	0.093	0.089

**Table 2:** Satisfaction after optimization of architectural landscape space.

Serial number	Evaluation factor	Square	Pedestrian street
1	Space security	0.43	0.29
2	Space privacy	0.76	0.32
3	Greening rate	0.84	0.66
4	Color diversity	0.58	0.35
5	Convenience of public facilities	0.85	052
6	A broad sense of vision	0.29	0.28
7	Leisure atmosphere	0.76	0.35
8	Individualization degree	0.59	0.42

RETRACTED

## Data Availability

The data that support the findings of this study are included within the article.

## References

[1] Jiang P., Fu Y. (2017). Research on the urban public art design and regional culture infiltration models in the background of Chinese urbanization. *Revista de la Facultad de Ingenieria*.

[2] Neto O. A., Munakata J., Jeong S. (2017). Public space design effect on users’ perceptions, impressions and intended activities. *Journal of Environmental Engineering*.

[3] Balint T. S., Pangaro P. (2017). Design space for space design: d. *Acta Astronautica*.

[4] Laing S., Apperley M. (2020). The relevance of virtual reality to communication design. *Design Studies*.

[5] David M., Follain S., Ciampalini R., Le Bissonnais Y., Couturier A., Walter C (2014). Simulation of medium-term soil redistributions for different land use and landscape design scenarios within a vineyard landscape in Mediterranean France. *Geomorphology*.

[6] Polat A. T., Akay A. (2015). Relationships between the visual preferences of urban recreation area users and various landscape design elements. *Urban Forestry and Urban Greening*.

[7] Verderber S. (2014). Residential hospice environments: evidence-based architectural and landscape design considerations. *Journal of Palliative Care*.

[8] Cai W., Liu D., Ning X., Wang C., Xie G. (2021). Voxel-based three-view hybrid parallel network for 3D object classification. *Displays*.

[9] Scognamiglio A., Garde F. (2016). Photovoltaics’ architectural and landscape design options for Net Zero Energy Buildings, towards Net Zero Energy Communities: spatial features and outdoor thermal comfort related considerations. *Progress in Photovoltaics: Research and Applications*.

[10] Wang J., Li F., Qian Y., Yin C. (2012). Landscape security pattern design based on ecosystem service. *Environmental Science & Technology*.

[11] Zhou Q. (2020). Research on architectural space design of coastal cities based on virtual reality technology. *Journal of Coastal Research*.

[12] Jaganmohan M., Knapp S., Buchmann C. M., Schwarz N. (2016). The bigger, the better? The influence of urban green space design on cooling effects for residential areas. *Journal of Environmental Quality*.

[13] Scorpio M., Laffi R., Masullo M. (2020). Virtual reality for smart urban lighting design: review, applications and opportunities. *Energies*.

[14] Sha C., Wang X., Lin Y., Fan Y., Chen X., Hang J (2018). The impact of urban open space and ‘lift-up’ building design on building intake fraction and daily pollutant exposure in idealized urban models. *Science of the Total Environment*.

RETRACTED

[15] Li J., Hou T. (2021). Application of virtual reality technology in analysis of the three-dimensional evaluation system of rural landscape planning. *Mathematical Problems in Engineering*.

[16] Allahyar M., Kazemi F. (2021). Effect of landscape design elements on promoting neuropsychological health of children. *Urban Forestry and Urban Greening*.

[17] Sun W., Yang X., Shan P. (2020). Research on ice and snow landscape design and visual aesthetic effect in coastal cold city. *Journal of Coastal Research*.

[18] Wang H. (2019). Landscape design of coastal area based on virtual reality technology and intelligent algorithm. *Journal of Intelligent and Fuzzy Systems*.

[19] Zhao M., Chang C. H., Xie W., Xie Z., Hu J. (2020). Cloud shape classification system based on multi-channel cnn and improved fdm. *IEEE Access*.

[20] Zhang J., Sun J., Wang J., Li Z., Chen X. (2022). An object tracking framework with recapture based on correlation filters and Siamese networks. *Computers & Electrical Engineering*.

[21] Chung A., To W. M., Schulte-Fortkamp B. (2016). Next generation soundscape design using virtual reality technologies. *Journal of the Acoustical Society of America*.

